The article "Loss of Cofilin 1 Disturbs Actin Dynamics, Adhesion between Enveloping and Deep Cell Layers and Cell Movements during Gastrulation in Zebrafish" was published in 2010. Journal: PLoS One.

# Loss of Cofilin 1 Disturbs Actin Dynamics, Adhesion between Enveloping and Deep Cell Layers and Cell Movements during Gastrulation in Zebrafish

**DOI:** 10.1371/journal.pone.0015331

**Published:** 2010-12-22

**Authors:** Chun-Wei Lin, Shuo-Ting Yen, Hui-Ting Chang, Shiang-Jiuun Chen, Shih-Lei Lai, Yi-Ching Liu, Tun-Hao Chan, Wen-Lian Liao, Shyh-Jye Lee

**Affiliations:** 1 Institute of Zoology, National Taiwan University, Taipei, Taiwan, Republic of China; 2 Department of Life Science, National Taiwan University, Taipei, Taiwan, Republic of China; 3 Institute of Fisheries Science, National Taiwan University, Taipei, Taiwan, Republic of China; 4 Center for Biotechnology, National Taiwan University, Taipei, Taiwan, Republic of China; Texas A&M University, United States of America

## Abstract

During gastrulation, cohesive migration drives associated cell layers to the completion of epiboly in zebrafish. The association of different layers relies on E-cadherin based cellular junctions, whose stability can be affected by actin turnover. Here, we examined the effect of malfunctioning actin turnover on the epibolic movement by knocking down an actin depolymerizing factor, cofilin 1, using antisense morpholino oligos (MO). Knockdown of *cfl1* interfered with epibolic movement of deep cell layer (DEL) but not in the enveloping layer (EVL) and the defect could be specifically rescued by overexpression of *cfl1*. It appeared that the uncoordinated movements of DEL and EVL were regulated by the differential expression of *cfl1* in the DEL, but not EVL as shown by in situ hybridization. The dissociation of DEL and EVL was further evident by the loss of adhesion between layers by using transmission electronic and confocal microscopy analyses. *cfl1* morphants also exhibited abnormal convergent extension, cellular migration and actin filaments, but not involution of hypoblast. The *cfl1* MO-induced cell migration defect was found to be cell-autonomous in cell transplantation assays. These results suggest that proper actin turnover mediated by Cfl1 is essential for adhesion between DEL and EVL and cell movements during gastrulation in zebrafish.

## Introduction

In the late gastrula stage, different types of cell migrations, including epiboly, involution, convergence, and extension, work together to form the embryonic germ layers and proper body structures [1], [2]. At this stage, a zebrafish embryo has three distinct cellular layers: the enveloping layer (EVL), deep cell layer (DEL) and yolk cell, which can be subdivided into the yolk cytoplasmic layer (YCL) and yolk syncytial layer (YSL) adjacent to the EVL. The EVL, a single-celled layer covering the mass of the DEL, has both tight junctions and filopodial activities with the YSL at its vegetal end as it undergoes epiboly [3], [4]. In concert with the EVL, the DEL also migrates toward the vegetal pole; and after the shield stage, part of the DEL, hypoblast, involutes at the margin into the space between the non-involuting DEL, epiblast, and yolk cell for a reverse anterior migration. The DEL then initiates convergence and extension movements before midgastrulation [5]. Both epiblast and hypoblast on the lateral side converge toward the dorsal side accompanied by their epibolic and involuting migration, respectively. Eventually, the dorsal-most portion of the DEL reaches the animal and vegetal poles.

The article "Loss of Cofilin 1 Disturbs Actin Dynamics, Adhesion between Enveloping and Deep Cell Layers and Cell Movements during Gastrulation in Zebrafish" was published in 2010. Journal: PLoS One.

The progression of the EVL margin towards the vegetal pole is at least in part dependent on the YSL by coupling to the EVL via tight junctions. Constriction of actin and myosin may be required to pull down the EVL [4]. Unlike the EVL, the molecular regulation of vegetal movement of DEL is less understood. A close association has been observed between DEL and EVL in an E-cadherin-dependent manner [6]. Thus the vegetal movement of DEL is presumably towing by EVL. This is supported by the arrest or delay of epiboly in DEL, but not EVL in zebrafish embryos lacking E-cadherin [6], [7], [8], [9]. These findings reveal that E-cadherin is required for the adhesion between DEL and EVL and this adhesion is essential for a proper DEL epibolic movement.

E-cadherin is the major transmembrane protein component of epithelial apical junctional complex (AJC), composed of tight junction (TJ) and adherens junction (AJ). By interacting with β-catenin and α-catenin, E-cadherin is coupled to actin filaments to consolidate the AJC [10]. The turnover of actin filament has been shown to affect the disassembly of AJC. We thus hypothesized that the actin filament turnover may also be involved in the E-cadherin-dependent association between DEL and EVL during gastrulation.

Highly active actin turnover occurs at the leading edge of motile cells. In a steady state, actin monomers polymerize at the barbed ends of actin filaments, and depolymerize from the pointed ends. Filament severing and nucleation both increase the numbers of barbed and pointed ends, thus promoting actin turnover and further protrusive activities [11]. Actin-depolymerizing factors (ADFs)/cofilins, one kind of actin-binding protein, can sever, stabilize, or nucleate actin filaments in a dosage-dependent manner [12]. They also were reported to be the primary factor enhancing actin turnover [13], [14], [15], and amplifying and specifying the direction of motile cells during chemotaxis [16]. These small (15∼21 kDa) ADFs/cofilins have conserved ADF-homology domains which are present in the closely related twifilins [17] and in some parts of several familiar proteins (e.g., drebrins) [18]. When a cofilin protein binds to an ATP-binding cleft on an actin filament helix, it changes the twist of the helix [19], and then bends the filament, thus accelerating actin filament severing [20]. But the ability to sever actin decreases as the concentrations of ADFs/cofilins increase [21], [22], [23]. That is, when the concentrations of ADFs/cofilins increase, actin filaments tend to be fully decorated by ADFs/cofilins resulting in a rather stabilized condition. And if the local ratio of ADFs/cofilins to actins increases, the actin tends toward nucleation.

The article "Loss of Cofilin 1 Disturbs Actin Dynamics, Adhesion between Enveloping and Deep Cell Layers and Cell Movements during Gastrulation in Zebrafish" was published in 2010. Journal: PLoS One.

ADFs/cofilins activities are directly activated by Slingshot phosphatase (SSH) [24] and inhibited by LIM kinase (LIMK) by dephosphorylation and phosphorylation on the N terminal serine 3 residue, respectively [25], [26]. Both SSH and LIMK are known downstream effectors of small GTPases [26], [27]. We have previously demonstrated the necessity of Rho signaling in mediating gastulation in zebrafish [28], [29]. In addition, the SSH was also been reported to play an essential role in *Xenopus* gastrulation [27]. Thus we reasoned that ADFs/cofilins may also be critical regulators in gastrulation by modulating actin turnover. However, in a large insertion mutagenesis screen, a zebrafish mutant harboring an insertion in the first intron of *cofilin 1* (*cfl1*) (previously known as *cofilin 2 like*) was identified and showed no obvious phenotype at one day after fertilization [30]. The lack of early gastrulation defect in zebrafish *cfl1* mutants is contradictory to previous studies described. It might be that the residual maternal *cfl1* messages presented in embryos were enough for the embryos to survive through early development. To clarify this issue, we have cloned the zebrafish *cfl1* and showed that *cfl1* is differentially expressed in DEL, but not in EVL in zebrafish embryos. We further demonstrated that the loss of *cfl1* induced by its respective morpholino results in the interference of epiboly, convergent extension, cell protrusions and directed cell migration during gastrulation.

## Results

### Sequence, syntenic, and structural analyses of zebrafish *cofilin 1*

In zebrafish, there are three homologous genes of ADF/cofilins: *cofilin 1* (*cfl1*, non-muscle form, AY398324), *cofilin 1-like* (*cfl1l*, AY398323) and *cofilin 2* (*cfl2*, muscle form, NM_205700). We were interested in cofilins, which are expressed during early embryogenesis and have the potential to regulate gastrulation cell migration. According to the available expression patterns in ZFIN, only *cfl1* and *cfl1l* fit into this category, as *cfl2* is mainly expressed in somites and later in myotomes and lenses. By a preliminary screening using an antisense morpholino oligo (MO), we found that knockdown of *cfl1l* had a minimum effect on gastrulation (our unpublished data). By contrast, the *cfl1* MOs showed severe interference with the progression of gastrulation (data will be described later). Thus, we had isolated the zebrafish *cfl1* gene by PCR cloning from zebrafish embryonic complementary DNAs. To compare its sequence identities and similarities of zebrafish Cfl1 to cofilins of other animal species, we aligned its amino acid sequence of with that of the non-muscle form of cofilins in mammals (including bovine, human, mouse, and rat), chick, western clawed frog, fish (including fugu and medaka), and the ADFs in the fruit fly (TSR) and nematode (UNC-60) (Fig. 1A). Zebrafish Cfl1 was highly similar to those cofilins examined (82%∼90%) except for the fruit fly (50%) and nematode (56%) (Fig. 1B). It was most similar to Cfl1 of medaka with 90% similarity. As shown in the phylogenetic tree (Fig. 1C), zebrafish Cfl1 was grouped together with the chordates, while the invertebrate ADFs (fly and nematode) were placed in an out-group cluster.

The article "Loss of Cofilin 1 Disturbs Actin Dynamics, Adhesion between Enveloping and Deep Cell Layers and Cell Movements during Gastrulation in Zebrafish" was published in 2010. Journal: PLoS One.

**Figure 1:** Sequence analysis of cofilin 1. (A) Amino acid sequences of zebrafish Cfl1 (**NP_998806**) was aligned with their orthologs of other species, including nematode (UNC-60, **NP_503427**), fruit fly (TSR, **NP_477034**), western clawed frog (xCfl1, **AAH67328**), bovine (bCFL1, **NP_001015655**), rat (rCFL1, **NP_058843**), human (hCFL1, **NP_005498**), mouse (mCFL1, NP_031713), fugu (fCfl1, **ENSTRUP00000031388**) and medaka (meCfl1, **ENSORLP00000002617**) using Vector NTI 10.3 software. Identical amino acids across all and some species are shaded in black and gray, respectively. (B) Similarity table of Cfl1 amino acid sequences of different species. (C) Phylogenic tree of Cfl1 amino acid sequences of different species. Both similarity tables and the phylogenic tree were generated by MEGA 4.0 software. (D) Syntenic analysis of zebrafish *cfl1* shows the similarity in chromosomal positions with human and mouse orthologs. (E) Sequence domain analysis of zebrafish Cfl1 with a putative phosphorylation site (P) and a nuclear localization sequence (NLS). The α-helices are shown in shaded boxes, and β-sheets are presented as open arrows. (F) Three-dimensional ribbon structure of Cfl1. N, N-terminus; C, C-terminus; NLS, nuclear localization sequence (boxed region with a red boundary).

To determine the chromosomal position of *cfl1*, we conducted a syntenic analysis of three cofilin genes (Fig. 1D). The *cfl1* in zebrafish, human, and mouse are located on chromosomes 14, 11, and 9, respectively. The same genes are found in the vicinity, which are *efemp2* (EGF-containing fibulin-like extracellular matrix protein 2) and *fibp* (fibroblast growth factor (acidic) intracellular binding protein), but zebrafish *cfl1* is arranged in a reversed orientation compared with those of human and mouse. These analyses suggest that zebrafish *cfl1* is evolutionarily related to mammalian cofilin 1 genes.

The article "Loss of Cofilin 1 Disturbs Actin Dynamics, Adhesion between Enveloping and Deep Cell Layers and Cell Movements during Gastrulation in Zebrafish" was published in 2010. Journal: PLoS One.

The primary amino acid sequence of Cfl1 contains 165 amino acids with a molecular weight of ∼18 kDa. The characteristic secondary structures are depicted in Fig. 1E. Cfl1 has six α-helices and seven β-sheets with a phosphorylation site at Ser 3 and a nuclear localization sequence (NLS, at residues 21∼38). A three-dimensional ribbon structure of Cfl1 created by SWISS-MODEL (http://www.swissmodel.expasy.org) is shown in Fig. 1F. Taken together, the zebrafish *cfl1* we isolated has high sequence and functional domain similarities compared to its orthologs from other species.

### Loss of Cfl1 interferes with epiboly movement

To further investigate the role of Cfl1 during embryogenesis in zebrafish, we separately injected embryos with two non-overlapping antisense MOs, tMO_1_ and tMO_2_ targeting the start codon and neighboring 5′-untranslated region (UTR) sequence of *cfl1* mRNA at −22 to +3 and −50 to −26, respectively, to block translation of *cfl1*. At 10 hours post fertilization (hpf), untreated embryos had completed epiboly and had entirely enclosed the yolk sphere (Fig. 2A). By contrast, knockdown of *cfl1* by tMO_1_ delayed or even arrested epiboly progression (Fig. 2B–C) in a dose-dependent manner and similar inhibition of epiboly was observed using the non-overlapping tMO_2_ (Table 1). Embryos injected with 10 ng tMO_1_, showed severe retardation in epiboly progression, and some of them could not complete gastrulation and ceased at about the 50% epiboly stage at 10 hpf (Fig. 2D). Embryos injected with lower tMO_1_ dosages had milder epiboly defects, most of them achieved 80%∼90% epiboly (Fig. 2C), and some of them only exhibited a malformed tail-bud (Fig. 2B). To further confirm that the severely retarded embryos are developmentally arrested, we monitored those 10 ng tMO_1_-injected embryos, which did not reach 100% epiboly at 10 hpf, until 12 hpf when the un-injected control embryos developed to 6-somite stage, and found that 235 out of 247 of those embryos (95.6±5.4%) still arrested at 60∼80% epiboly in three trials.

**Figure 2:** Knockdown of *cfl1* causes epiboly defects. Embryos were injected with or without *cfl1* MO and photographed at 10 h post-fertilization (hpf). The *cfl1* MO caused epiboly defects of different severities. (A) A sham-injected embryo reached 100% epiboly. (B) A *cfl1* morphant with a malformed tail bud. (C) A *cfl1* morphant that reached 90% epiboly. (D) A *cfl1* morphant that reached 50% epiboly. Scale bar, 200 µm.

The article "Loss of Cofilin 1 Disturbs Actin Dynamics, Adhesion between Enveloping and Deep Cell Layers and Cell Movements during Gastrulation in Zebrafish" was published in 2010. Journal: PLoS One.

**Table 1:** Loss of Cfl1 dose-dependently causes epiboly defect.

Treatments	% of epiboly defect	Number of embryos
Sham-injected	4.9±2.0^a^	98
tMO_1_ (ng/embryo)		
2.5 ng	10.7±2.0^a^	118
5.0 ng	65.6±2.9^b^	107
7.5 ng	78.7±4.5^c^	112
10 ng	81.9±4.4^c^	100
Sham-injected	5.5±4.7^a^	129
tMO_2_ (ng/embryo)		
2.5 ng	34.5±31.5^b^	113
5.0 ng	63.9±25.8^c^	123
7.5 ng	90.6±8.8^c^	106
10 ng	88.7±7.8^c^	122

*Note*: Embryos at 1-cell stage were injected without (sham-injected with 2.3 µL injection buffer) or with different dosages of *cfl1* tMO_1_ or tMO_2_ and examined at 10 hpf. Some embryos died (usually <10%) at 10 hpf and were not counted in these experiments. Embryos did not reached 100% epiboly were considered to have epiboly defect. These experiments were repeated 4 times. Data are presented as means ± standard deviation. Experimental values are compared within groups, subjected to ANOVA and the mean separation was done by Duncan's Multiple Range Test (DMRT). Values with different lettering in their superscripts are significantly (p<0.05) from each other.

To examine whether the zygotic Cfl1 expression can be inhibited by *cfl1* MOs, we inserted a stretch of *cfl1* nucleotides ∼200-bp, which contains their respective MO target site, into a pCS2+ XLT vector with a green fluorescent protein (GFP) gene and co-injected these constructs with their respective MO. Embryos (81.0±13.8%) injected with the pCS2+ XLT with tMO_1_ binding site (tMO_1_ plasmid) expressed GFP fluorescence (Fig. 3A). By contrast, none of embryos co-injected with tMO_1_ showed GFP fluorescence (Fig. 3B). Similarly, embryos (79.4±11.9%) injected with the pCS2+ XLT with tMO_2_ binding site (tMO_2_ plasmid) expressed GFP fluorescence, but not in those embryos co-injected with tMO_2_ (Fig. 3C). Both MOs appeared to be equally effectively, we thus used tMO_1_ for the rest of experiments unless otherwise stated.

**Figure 3:** *Cfl1* MOs efficiently block the translation of GFP fusion constructs containing respective MO binding site. Embryos at 1-cell stage were injected with 330 pg pCS2+ XLT fused with a fragment of *cfl1* gene sequence from −22 to +195 or −52 to +51 in the absence or presence of 7.5 ng *cfl1* tMO_1_ or tMO_2_, respectively. The expression of GFP was examined at 10 hpf and photographed under epifluorescent microscopy. The representative photos for embryos treated without *cfl1* MO (A) and with tMO_1_ (B) are shown and the percentages of injected embryos expressing GFP are shown in average ± standard deviation (C).

The article "Loss of Cofilin 1 Disturbs Actin Dynamics, Adhesion between Enveloping and Deep Cell Layers and Cell Movements during Gastrulation in Zebrafish" was published in 2010. Journal: PLoS One.

To confirm that the defects we observed in *cfl1* morphants were specifically due to the loss of Cfl1 activity, we examined whether overexpression of *cfl1* could rescue the *cfl1* morphant defects. *cfl1* was successfully overexpressed as revealed by the presence of GFP fluorescence in zebrafish embryos injected with mRNAs prepared from a PCS2+ XLT vector containing the full *cfl1* coding sequence (data not shown). More importantly, the inhibition of epiboly could be significantly (P<0.05) reduced in embryos co-injected with 100 pg *cfl1-egfp* mRNAs and 7.5 ng tMO_1_ (Table 2). Furthermore, depending on the sequence specificity of MOs, MOs may have caused secondary effects like p53-dependent apoptosis [31]. To examine whether the effect of the *cfl1* MO was mediated by p53, we co-injected the *cfl1* tMO_1_ (7.5 ng) with a p53 MO (7.5 ng) into zebrafish embryos and found that both epiboly progression and mortality of co-injected embryos did not significantly (P>0.05) differ from those embryos injected with only the *cfl1* tMO_1_ (Table 2).

**Table 2:** Cfl1 MO-induced epiboly defect can be partially rescued by co-injection of *cfl1* mRNA, but not P53 MO.

Treatments	Bud (%)	90% epiboly (%)	75% epiboly (%)	Death (%)	Number of embryos
StdMO	97.0±4.2^a^	0.8±1.7^a^	0.0±0.0^a^	2.2±4.4^a^	149
tMO_1_	9.7±6.8^b^	28.6±14.2^b^	53.3±26.4^b^	8.4±9.6^a^	166
tMO_1_ + *cfl1* mRNA	49.6 ±11.8^c^	36.9±7.7^b^	8.7±10.7^a^	4.8±4.0^a^	160
Un-injected	96.6±4.0^a^	0.7±1.3^ a^	1.3±2.6^ a^	1.4±2.8^ a^	178
tMO_1_	0.0±0.0^ b^	7.9±10.7^ b^	84.8±9.0^ b^	7.3±4.8^ b^	145
tMO_1_ + p53 MO	0.6±1.2^ b^	7.9±7.5^ b^	78.5±14.3^ b^	13.0±10.6^ b^	145

*Note*: Embryos at 1-cell stage were injected with *cfl1* tMO_1_ (7.5 ng per embryo) without or with *cfl1* mRNA (100 pg per embryo) or p53 MO (7.5 ng per embryo) and examined at 10 hpf. The percentages of epiboly progression were recorded. These experiments were repeated 4 times. Data are presented as means ± standard deviation. Experimental values are compared within groups, subjected to ANOVA and the mean separation was done by Duncan's Multiple Range Test (DMRT). Values with different lettering in their superscripts in the same column of each group are significantly (p<0.05) from each other.

### *cfl1*-tMO_1_ causes unsynchronized migration of EVL and DEL and over-polymerization of filamentous actin

To examine the effects of *cfl1* knockdown on the actin cytoskeleton structure, the filamentous actin (F-actin) was stained by rhodamine phalloidin, and to better differentiate individual cells nuclei were visualized by a nuclear dye DAPI (4′,6-diamidino-2-phenylindole). The double-stained embryos were examined under confocal microscopy (Fig. 4). At the lower magnification, the margins of EVL and DEL did not appear to migrate together during epiboly in *cfl1* morphants (Fig. 4D) compared to the synchronized movements in control embryos (Fig. 4A). At a higher magnification, it clearly showed that the EVL was 2 or 3 rows of cells ahead of the DEL (Fig. 4E, F). This uncoordinated migration between the EVL and DEL was even more obvious in embryos injected with a higher dosage (10 ng) of *cfl1*-tMO_1_ (data not shown). At the higher magnification, the YSL actin cable (arrow) and cell boundary actin were notably intense and condensed in *cfl1* morphants (Fig. 4E) compared to control embryos (Fig. 4B).

The article "Loss of Cofilin 1 Disturbs Actin Dynamics, Adhesion between Enveloping and Deep Cell Layers and Cell Movements during Gastrulation in Zebrafish" was published in 2010. Journal: PLoS One.

**Figure 4:** Knockdown of *cfl1* enhances the filamentous actin (F-actin) formation and attenuates adhesion between the EVL and the DEL. Embryos at the 65%∼70% epiboly stage were fixed, stained with rhodamine phalloidin and DAPI to reveal F-actin and nuclei, respectively, under confocal microscopy. Confocal images of whole-embryo sections at a lower magnification are shown for untreated (A) and *cfl1* tMO_1_-injected embryos (B). In the untreated embryo (A), an arrow indicates synchronous leading edges of EVL and DEL whereas distinctly separated leading edges are obvious as pointed by arrows in *cfl1* tMO_1_-injected embryos (B). At a higher magnification (B, C, E, F), F-actin was more condensed at the boundaries of blastomeres and the margin of blastoderm (arrows) of *cfl1* morphants (E) compared to untreated embryos (B). The progression of the EVL margin (arrow) was more advanced than that of DEL (dashed line) in *cfl1* morphants (E) compared to that of untreated embryos (B). From the side view (C, F), the EVL margin (upper arrow) was clearly advanced 2 cells ahead of DEL (lower arrow) in *cfl1* morphants (F) that was not seen in untreated embryos (C). Scale bars: 25 µm for A and D; 250 µm for B, C, E, F.

### Temporal and spatial expression profile analyses of *cfl1*

The unsynchronized movements of EVL and DEL in *cfl1* morphants led us to suspect that *cfl* may be expressed differentially and result in different responses upon knockdown of *cfl1*. The RT-PCR analysis showed that *cfl1* was expressed throughout development and was present in all adult tissues examined (data not shown). To gain the temporal and spatial profiles of *cfl1* during embryogenesis, we thus performed whole-mount *in situ* hybridization (WISH) in different stages of embryos (Fig. 5). The WISH analysis revealed that the expression domains of *cfl1* during early development were ubiquitous until the sphere stage (Fig. 5A–D). The *cfl1*'s expression was notably reduced at 30% epiboly (Fig. 5E) and the shield stages (Fig. 5F), and it was absent from the future ventral side of the embryo in the bud stage (Fig. 5G). *cfl1* was strongly expressed throughout the embryo body during early segmentation period (Fig. 5H); it was later restricted to the central nervous system, lateral line, and pronephric duct at 26∼31 hpf (Fig. 5I and J); and expression domains were evident in the brain, pharyngeal arches, lateral line, and pronephric duct in the larval stages (3∼5 days post-fertilization, Fig. 5K–N). We were in particular interest in the expression of *cfl1* at different cell layers of a gastrulating embryo, thus we performed cryo-section for those 70% epiboly stage embryos underwent WISH against *cfl1*. Interestingly, we found that the *cfl1* expression domain was restricted to blastomere boundaries of the DEL, but not those of the EVL (Fig. 5O).

The article "Loss of Cofilin 1 Disturbs Actin Dynamics, Adhesion between Enveloping and Deep Cell Layers and Cell Movements during Gastrulation in Zebrafish" was published in 2010. Journal: PLoS One.

**Figure 5:** Spatial and temporal expression of *cfl*1 during embryogenesis. (A–N) Representative whole-mount *in situ* hybridization photographs are shown to reveal the expression patterns of *cfl1* at the designated stages from 1-cell to 5 day post-fertilization (dpf) as denoted at the lower left corner of each panel. (O) A representative cryo-section photograph of an embryo at the 70% epiboly stage underwent WISH against *cfl1*. The cryo-section was taken from the box region as depicted in the embryo carton shown on the right. b, brain; ba, bronchial arches; ll, lateral line system; pd, pronephric duct; pa, pharyngeal arches; EVL, enveloping layer; DEL, deep cell layer. Scale bars: 400 µm for the 4- and 5-dpf embryos, 200 µm for the others and 50 µm for the cryo-section photograph.

### Loss of Cfl1 retards vegetal migration in the DEL but not the EVL

It is known that a close contact association exists between EVL and DEL [6]. We therefore examined whether the unsynchronized movements of EVL and DEL is due to the loss of their association by transmission electron microscopy (TEM). Clear disruptions of EVL-DEL attachments were observed in *cfl1* morphants as evidenced by spaces in part of the contact zones between the DEL and EVL (Fig. 6B) compared to that in control embryos (Fig. 6A).

**Figure 6:** Loss of Cfl1 causes disruption of the attachment between the EVL and DEL. Embryos injected with either the StdMO (A) or c*fl1* tMO_1_ (B) were fixed at 8.5 hpf and subjected to transmission electron microscopy. Cohesive attachment between the EVL and DEL on lateral sites of embryos was observed in StdMO-treated control embryos, but a cleft (aster) was observed in *cfl1* morphants. Each photograph is representative of at least five embryos with similar results.

The article "Loss of Cofilin 1 Disturbs Actin Dynamics, Adhesion between Enveloping and Deep Cell Layers and Cell Movements during Gastrulation in Zebrafish" was published in 2010. Journal: PLoS One.

To further compare dynamic interactions between the DEL and EVL, we performed live imaging analysis of a gastrulating embryo from 7.5 to 8.5 hpf under confocal microscopy. We focused on the dorsolateral sites of embryos injected with membrane-bound GFP-GAP43 mRNAs and the StdMO or *cfl1* tMO_1_. While both the DEL and EVL showed highly coordinated migration toward posterior sites in control embryos (Fig. 7, left column; Supplementary Movie S1), cells of the DEL in *cfl1*-morphants did not form tight attachments and showed a clear gap with EVL cells (Fig. 7, right column; Supplementary Movie S2). In addition, a very dynamic change in cell shape was observed in DEL cells of control embryos, but not in those of *cfl1* morphants (Supplementary Movie S2).

**Figure 7:** Live cell imaging reveals loose cell-cell interactions between the DEL and EVL in c*fl1* morphants. Embryos injected with designated MOs and membrane-bound green fluorescent protein (GFP) mRNA, were dechorionated, immobilized, and examined by confocal microscopy for 10-min recordings at 10-s intervals per frame. The snapshots of representative embryos from the StdMO- (left column) or *cfl1*MO-injected embryos (right column) are shown. The recording times in minutes are denoted in the lower left corner of the left column. While StdMO-treated embryos showed continuous tight attachments between the DEL and EVL, DEL cells in *cfl1* morphants did not form a tight connection with the EVL, which was further evidenced by the more-rounded cell shapes. Arrowheads indicate spaces between the EVL and DEL. A single-cell-thick EVL is to the right; yolk cells are toward the left; the animal pore is on the top; and the vegetal pore is at the bottom.

### Loss of Cfl1 perturbs convergent extension but not involution during gastrulation

To further investigate how Cfl1 affects cell movements during gastrulation, we conducted cell tracing assays using caged Q-rhodamine dextran [32]. Caged Q-rhodamine was injected with or without the *cfl1* tMO_1_ into one-cell stage embryos and later uncaged by brief exposure to ultraviolet light to mark a selected group of cells. To monitor dorsal convergence movements, we marked cells in the lateral blastoderm margin at 90° from the dorsal embryonic shield, and fluorescent cells were traced during gastrulation. The marked cells in the control StdMO-injected embryos moved dorso-anteriorly, and had extended along the anterior-posterior (AP) axis at 10.5 hpf (Fig. 8A, upper panels), as previously reported [33], [34]. By contrast, the anterior migration and convergence of lateral mesendodermal cells toward the dorsal side were notably impaired in *cfl1* morphants (Fig. 8A, lower panels). Measuring the degree of convergence (θ =  sin^−1^(r/R)) from the origin of the marked cells in control and treated embryos at different times after recording and plotting the results against the time (hpf) showed that the fitted slope of *cfl1* tMO_1_-injected embryos (y = 10.7x - 69.7) clearly deviated from that of StdMO-injected ones (y = 15.6x - 96.2) (Fig. 8C). To examine the effect of *cfl1* tMO_1_ on AP extension movements, cells of dorsal embryonic shields were marked and monitored as previously described in StdMO- and *cfl1* tMO_1_-injected embryos (Fig. 8B). In control StdMO-injected embryos, marked cells were found in the dorsal axial hypoblast along the entire AP axis at 10.5 hpf (Fig. 8B, upper panels) which is consistent with a previous report [34]. By contrast, the anterior movement of marked cells was perturbed, exhibiting a shortened axial mesoendoderm in *cfl1* tMO_1_-injected embryos (Fig. 8B, lower panels). Measuring the angle (ϕ) between two arrows of the anterior and posterior ends of the marked axial mesoendoderm connecting to the center of the embryos (Fig. 8B) in control and treated embryos at different times after recording and plotting the results against times of measurement demonstrated that the fitted slope (33.2x - 215.8) of *cfl1* tMO_1_-injected embryos was also lower than that of StdMO-injected ones (y = 41.7x - 261.9) (Fig. 8D). Furthermore, we also conducted WISH to reveal the anterior edge of the neural plate and prechordal plate by probing against *cathepsin L 1 b* (*cstl1b*) and *distal-less homeobox gene 3b* (*dlx3b*), respectively. The body axis was severely shortened and broadened in tMO_1_-treated embryos (Fig. 8E) compared to that of control embryos (Fig. 8F).

The article "Loss of Cofilin 1 Disturbs Actin Dynamics, Adhesion between Enveloping and Deep Cell Layers and Cell Movements during Gastrulation in Zebrafish" was published in 2010. Journal: PLoS One.

**Figure 8:** Knockdown of *cfl1* causes convergent and extension defects. (A, B) Embryos were injected with Q-rhodamine with or without *cfl1* tMO_1_ and incubated in the dark. Cells of the lateral (A) and dorsal blastomere margins (B) are marked as shown in red fluorescence at the shield stage and observed until 10.5 hpf. Representative photographs taken at 6.5, 8.5 and 10.5 hpf for both the untreated control and *cfl1* MO-injected embryos are shown. (C) As shown in the panel A with an 8.5-hpf control embryo, the radius of the embryo (R) and the migration distance of the labeled cells (r) were measured. The degree of convergence (θ) was calculated by applying the following equation: θ =  sin^−1^(r/R), and then plotted against the stage of the embryo in hpf. (D) As shown in panel B with an 8.5-hpf control embryo, the angle (φ) between the two arrows of the anterior and posterior ends of the marked axial mesoendoderm connecting the center of the embryo was measured in each embryo to estimate the degree of extension. The degree of extension (φ) was then plotted against the stage of the embryo. (E, F) WISH against *cstl1b* (expressed in the prechordal plate as indicated by asterisks) and *dlx3b* (expressed in paraxial mesoderm as indicated by arrows) of bud-stage zebrafish embryos was performed. Representative photographs in frontal view are shown for an untreated (E) and a *cfl1* tMO_1_-injected embryo (F).

To examine whether the internalization of epiblast (i.e. involution) was affected by the reduction of *cfl1* translation, we have treated embryos with 5.0 or 7.5 ng of tMO_1_ or stdMO, fix and subjected them to WISH against *cstl1b*. The appearance of *cstl1b* is an indication of formation of prechordal plate and thus the occurrence of involution. In two independent trials, involution occurred in all embryos treated with both dosages of tMO_1_ tested (Fig. 9A–F for 7.5 ng, n = 46; Fig. 7G–L for 5 ng, n = 49) as those embryos injected with stdMO (Fig. 9M–R, n = 55).

**Figure 9:** Knockdown of *cfl1* does not affect involution of mesendoderm. Embryos injected with 7.5 ng Std MO (A–F), 5.0 ng (G–L) or 7.5 ng *cfl1* tMO_1_ (M–R) were examined at 10 hpf (A, B, G, H, M, N), fixed and subjected to WISH against *cstl1b* (C–F, I–L, O–R). Representative photographs were taken at a lower (6.3X) or higher (50X) magnification and scale bars are shown at the bottom panel of each column (1 mm for 6.3X and 200 µm for 50X).

### Cfl1 mediates pseudopod formation of involuting cells in a cell-autonomous manner

Cellular migration requires actin-based pseudopod extensions in which Cfl1 might participate. To examine the role of Cfl1 in the formation of pseudopods during gastrulation, we applied time-lapse recording to monitor dynamic changes in migrating cells during the 75%∼90%-epiboly stages by targeting the apparent margins of involuting cells. After the germ-ring stage, both lateral (mesendodermal cells) and prechordal plate cells (progenitor cells) began involution from a lateral or dorsal site, respectively. Concomitantly, lateral cells converged toward the dorsal site while prechordal plate cells extended to the anterior. During a 15-min time-lapse recording, StdMO-injected embryos formed a normal number of pseudopods per cell in both lateral cells (6.7±1.1, Supplementary Movie S3) and prechordal plate cells (6.6±1.1, Supplementary Movie S5). By contrast, the number of pseudopods per cell in *cfl1* tMO_1_-injected embryos was significantly (*p*<0.05) lower in both lateral cells (2.8±0.8, Supplementary Movie S4) and prechordal plate cells (3.5±0.5, Supplementary Movie S6). Representative images are shown in Fig. 10A–D, and the average number of protrusions formed in each treatment is presented in Fig. 10E.

The article "Loss of Cofilin 1 Disturbs Actin Dynamics, Adhesion between Enveloping and Deep Cell Layers and Cell Movements during Gastrulation in Zebrafish" was published in 2010. Journal: PLoS One.

**Figure 10:** Knockdown of *cfl1* inhibits the pseudopod formation of involuting cells. Embryos injected with MOs were dechorionated, immobilized, monitored, and recorded in 15-min continuous time-lapse movies. Lateral cells were monitored from the lateral side (A, C), and prechordal plate cells were monitored from the anterior side (B, D). Representative photographs are shown for each group as designated. Arrows indicate the sites of pseudopods. (E) Number of pseudopods was counted and analyzed for each group. Both lateral cells and prechordal plate cells in *cfl1* morphant embryos had significantly fewer pseudopods (* *p*<0.05). Only upper error bars of the standard deviations are shown.

To further evaluate the cell autonomy of Cfl1 functions, cells from embryos injected with MOs and rhodamine-dextran, were transplanted into untreated host (control) embryos and *cfl1* morphants respectively. Only those transplanted cells undergoing epiboly were selected for further analysis. The protrusive activities of these transplanted cells were examined by confocal microscopy, and representative snapshots were taken to show the polygonal shape and pseudopod formation by StdMO-injected cells in control hosts (arrow heads in Fig. 11A; Supplementary Movie S7) and in *cfl1* morphants (Fig. 11C; Supplementary Movie S8), while *cfl1* tMO_1_-injected cells remained rounded with blebbing-like structures in control hosts (arrow in Fig. 11B; Supplementary Movie S9) and in *cfl1* morphants (Fig. 11D; Supplementary Movie S10). Furthermore, to reveal the migration velocity and direction of movement, we took time-lapse recordings under an epifluorescence microscope to trace cells from both StdMO- and *cfl1* MO-injected embryos transplanted into untreated or *cfl1* morphants. After analysis, we found that both the exact velocity (Vcl: curvilinear velocity; curvilinear distance/time) and directed velocity (Vsl: straight line velocity; straight line distance/time) were significantly reduced in *cfl1* tMO_1_-injected cells compared to StdMO-injected cells when transplanted into an untreated host embryo (Fig. 11E). This indicates that cofilin functions cell autonomously in transplanted cell migration. In the same logic, both Vcl and Vsl of *cfl1* tMO_1_-injected cells significantly reduced when transplanted into *cfl1* morphants. However, the Vcl and Vsl of StdMO-injected cells is also significantly reduced when transplanted into *cfl1* morphants, although was not as severe as *cfl1* tMO_1_-injected cells in the same background (Vsl, Fig. 11E).

The article "Loss of Cofilin 1 Disturbs Actin Dynamics, Adhesion between Enveloping and Deep Cell Layers and Cell Movements during Gastrulation in Zebrafish" was published in 2010. Journal: PLoS One.

**Figure 11:** Cfl1 is required cell-autonomously for proper epiboly cell migration. Labeled cells from donor embryos injected with rhodamine-dextran in combined with StdMO (**A,** **C**) or *cfl1* tMO_1_ (B, D) were transplanted into control embryos (A, B) and *cfl1* morphants (C, D) respectively, and recorded under a confocal microscope. Pseudopods (arrowheads) and polygonal cell shape were observed in StdMO-injected cells transplanted in both control hosts (A) and *cfl1* morphants (C), while blebbing-like structure (arrows) and rounded cell shape were observed in *cfl1* tMO_1_-injected cells transplanted in both control hosts (B) and *cfl1* morphants (D). The photographs shown are representative of at least 10 embryos in each experiment. Migration curvilinear velocity (Vcl) and straight line velocity (Vsl) of these StdMO- and *cfl1* tMO_1_-injected cells in control hosts or *cfl1* morphants were recorded by time-lapse epifluorescent microscopy and analyzed by SimplePCI software, respectively (E). Values between groups were compared using unpaired Student's *t*-test, and those showing a significant (* *p*<0.05) difference are denoted by different letters.

## Discussion

We have previously demonstrated that Rho mediates gastrulation cell movements in zebrafish via Rho-associated kinase [29] and Diaphanous [28], by regulating the contractile activity of actin filaments. Herein, we further delineated an essential role of a Rho downstream effector, cofilin, in zebrafish gastrulation by demonstrating the inhibitions of epiboly, convergence, and extension, but not involution by knocking down *cfl1*. The effects of *cfl1* knockdown were shown to be cell-autonomous and presumably via affecting actin turnover as evident by the over-polymerization of F-actin seen in *cfl1* morphants. The *cfl1* MOs also inhibited coordinated movement of EVL and DEL due to the disruption of their attachments and cellular contacts between two layers.

The uncoordinated movements between the EVL and DEL observed in *cfl1* morphants (Fig. 4) has been reported in E-cadherin-deficient embryos [6], [7], [8], [9]. Tight adhesion between the DEL and EVL is known to be exerted by E-cadherin mediated AJC that presumably allows the towing of DEL toward vegetal pole during gastrulation [6]. To examine whether the uncoordinated movement between the EVL and DEL was due to the disrupted EVL-DEL association, we showed the physical disruption of EVL/DEL attachment in *cfl1* morphants by TEM analysis (Fig.6) and time-lapse cellular recording (Fig. 7 and supplementary Movie S2). Because actin turnover is critical for maintaining AJC [35], thus Cofilin 1 may be required for the E-cadherin-mediated adhesion of EVL/DEL. Furthermore, cryo-sections of *cfl1*-WISH-labeled embryos showed restricted *cfl1* mRNA signals in the DEL but not the EVL at the 70% epiboly stage (Fig. 5). This differential expression of *cfl1* suggests that Cfl1 might only function in the DEL. Indeed, we clearly demonstrated that loss of Cfl1 only hampered movement of the DEL but not the EVL (Fig. 4,7). Although the EVL was shown to have filopodial activities toward the YSL [3], the lack of *cfl1* expression suggests that its filopodial activities may be regulated by factors other than Cfl1. In addition, tight junctions which exist between the EVL and YSL might passively drive epibolic migration of the EVL epiboly [4]. With intact DEL-EVL association, the DEL can be towed by the EVL during epiboly. However, this interaction between DEL and EVL was apparently lacking in *cfl1* morphants, which might have resulted in the uncoordinated migration.

The article "Loss of Cofilin 1 Disturbs Actin Dynamics, Adhesion between Enveloping and Deep Cell Layers and Cell Movements during Gastrulation in Zebrafish" was published in 2010. Journal: PLoS One.

The clear separation of margins of the DEL and EVL in *cfl1* morphants (Fig. 4,6B,7) suggests that cell-cell interactions between the DEL and EVL were affected. This pathological phenomenon is similar to that seen in E-cadherin (cadherin 1, *cdh1*)-deficient embryos [6], [7], [8], [36]. DEL-EVL but not DEL-DEL or EVL-EVL cell attachments were disrupted in both *cfl1* and *cdh1* knockdown embryos. E-cadherin interacts with actin cytoskeleton by a complex with β-catenin which binds to the actin-binding protein α-catenin [37], [38]. These serial bindings may stabilize the membrane-bound *cdh1* and form tight cell adhesions in these adherent junctions. It might be possible that knockdown of *cfl1* reduces actin turnover, disrupts the proper structures of actin filament networks in the DEL near the contact regions with the EVL, and results in unstable membrane-bound *cdh1* and abnormal detachments from the EVL. Unlike the EVL, the force driving the DEL to undergo epiboly is still unclear. However, active cell protrusions between the DEL and EVL at the margins of the epiboly were observed in wild-type zebrafish embryos [39]. These active cellular protrusions may assist in maintaining the tight interaction between the DEL and EVL. Thus, EVL could lead the DEL towards the vegetal pole to complete the epiboly. It is clear that the differential expression of *cfl1* in the DEL but not in EVL (Fig. 5O) allowed us to disrupt this interaction by simply knocking down *cfl1* activity in DEL and further demonstrated the importance of proper interaction of both layers in epiboly progression.

ADF/Cofilin has recently been suggested to play a functional node in cell biology [40]. Recently, it has been found that instead of its conventional role in actin depolymerization, cofilin can either promoting actin filament assembly or disassembly depending on their cellular concentrations and their ration to actin and other actin binding proteins [41]. It can also compete for actin at actin branches with ARP2/3 [42], which is known to be critical actin branches during embryogenesis [43], [44], [45], [46], [47]. Cofilin also contains functions unrelated to actin. It has been suggested to chaperon actin, which is lacking nuclear location signal, into nucleus [40], Upon cell stress, it can be translocated to mitochondrial [48] to induce the release of cytochrome c and subsequent apoptosis [49], [50]. The phospho-cofilin can directly activate phospholipase D (PLD) [51], which can mediates chemotaxis [52] and membrane lipid metabolism. It certainly deserves further investigations to determine whether cofilin exerts its effects on gastulation cell movements via any of its above-described novel functions in addition to the control of actin dynamics.

The article "Loss of Cofilin 1 Disturbs Actin Dynamics, Adhesion between Enveloping and Deep Cell Layers and Cell Movements during Gastrulation in Zebrafish" was published in 2010. Journal: PLoS One.

The lack of early phenotype in *cfl1* insertion mutants in zebrafish [30] is puzzling and contradictory to the necessity of cofilin as demonstrated in *Xenopus* embryos [27]. In this study, we demonstrated that Cfl1 is also essential for proper gastrulation cell movements in a cell-autonomous manner by mediating actin dynamics. Its differential expression in the EVL and DEL, and different migration patterns of the EVL and DEL in *cfl1* morphants further suggest that differential actin regulation is necessary to maintain adhesion of embryonic layers for cohesive epibolic movement in zebrafish. The lack of gastrulation defect observed in *cfl1* mutants is presumably due to the presence of maternal *cfl1* that helps the mutant embryos pass the gastrulation process.

## Materials and Methods

### Ethics Statement

All animal handling procedures were approved by the use of laboratory animal committee at National Taiwan University, Taipei, Taiwan (IACUC Approval ID: 97 Animal Use document No. 55).

### Zebrafish maintenance and embryo culture

Wild-type zebrafish (AB/TU) were raised under a 14-h light/10-h dark cycle at 28.5°C. Embryos were collected at 15∼20-min intervals after spawning, washed, and incubated in 0.3x Danieau's buffer (by diluting 1x Danieau's buffer consisting of 58 mM NaCl, 0.7 mM KCl, 0.4 mM MgSO_4_, 0.6 mM Ca(NO_3_)_2_, and 5.0 mM HEPES (pH 7.6) with double-distilled water) supplemented with 50 µg/mL streptomycin and 50 µg/mL penicillin G at 28.5°C until observation or fixation.

### Morpholino oligonucleotides (MOs) and mRNA preparation

Antisense MOs were purchased from Gene Tools (Philomath, OR) or Open Biosystems (Huntsville, AL). The standard MO (StdMO; sequence: 5′-CCTCTTACCTCAGTTACAATTTATA-3′) without sequence homology to any known zebrafish DNA sequences was used as a control treatment. To knock down zebrafish *cfl1* expression, two translational-blocking MOs (tMO), tMO_1_ (targeting the start codon and neighboring 5′-untranslated region (UTR) sequence of *cfl1* mRNA, −22 to +3; sequence: 5′-CATGGCTGTGTCTCTGTGCTAGTCG-3′) and tMO_2_ (targeting 5′-UTR sequences of *cfl1* mRNA, −50 to −26; sequence: 5′-TCTGGGTTGGAATTGAATGAGCTGT-3′) were used. To counter p53 activity, a p53 MO (sequence: 5′-GCGCCATTGCTTTGCAAGAATTG-3′) was used. To examine the translation blocking efficiency of *cfl1* tMO_1_ and tMO_2_, two pCS2+ XLT constructs were generated with an insertion of *cfl1* gene fragmen from −43 to +189 and −52 to +51, respectively. The *cfl1* tMO_1_ and tMO_2_ were co-injected with respective pCS2+ XLT plasmid and the % of embryos expressing GFP fluorescence was determined. To prepare *cfl1* expression vector, the full coding region of *cfl1* was inserted into pCS2+ XLT vector, which contains the green fluorescent protein (GFP) sequence following the insertion site. The *cfl1*-*gfp* construct was linearized by *Not*I, and the capped RNA was transcribed according to the manufacturer's instruction using a mMESSAGE mMACHINE® SP6 Kit (Applied Biosystems, Foster City, CA 94404).

The article "Loss of Cofilin 1 Disturbs Actin Dynamics, Adhesion between Enveloping and Deep Cell Layers and Cell Movements during Gastrulation in Zebrafish" was published in 2010. Journal: PLoS One.

### Microinjection procedures

Glass capillaries (1.14×0.50 mm, O.D. × I.D., World Precision Instrument, Sarasota, FL) were pulled using a horizontal puller (P-97, Sutter Instrument, Navato, CA). Embryos were collected after spawning, and then immobilized by an injection trough on a 100-mm 1% agar plate. An injection pipette was forced through the chorion, into the yolk cell and reached the area adjacent to the blastomeres where 2.3–4.6 nL of the desired solution was ejected using a Nanoliter injector (World Precision Instrument). Before injection, all solutions were diluted by 1x Danieau's buffer with phenol red (0.25% (w/v), pH 7.4) to the desired concentrations. Microinjection was completed before the embryos had reached the 4-cell stage. After injection, embryos were recovered from the trough and cultured at 28.5°C for further experiments.

### Whole-mount in situ hybridization (WISH) and cryosection

Embryos injected with MOs were grown in 0.3x Danieau's buffer supplemented with 0.2 mM 1-phenyl-2-thiourea (Sigma) to inhibit pigment formation [53], fixed at the desired developmental stages with 4% fresh paraformaldehyde in phosphate-buffer saline (PBS) overnight. After being manually dechorionated with fine forceps, embryos then transferred and stored into 100% methanol at −20°C. WISH was performed according to Thisse et al. [54], [55] using a DIG-labeled, SP6-RNA polymerase-made riboprobes hybridized to *cfl1* or *cfl1l*. For cryosections, stained samples were immersed in PBS containing 30% sucrose overnight, and embedded in Optimal Cutting Temperature (OCT) compound embedding medium (Sakura, Tokyo, Japan) at −20°C, and 10-µm frozen cross-sections were cut with a CM 1900 rapid sectioning cryostat (Leica, Heidelberg, Germany) and attached to poly-L-lysine-coated slides (Electron Microscopy Sciences, Ft. Washington, PA). Stained embryos and sections were observed under a stereomicroscope (Mz75, Leica Microsystems) and a DM5000B DIC system, respectively. Photographs were taken using a digital camera (Coolpix 995, Nikon, Melville, NY).

The article "Loss of Cofilin 1 Disturbs Actin Dynamics, Adhesion between Enveloping and Deep Cell Layers and Cell Movements during Gastrulation in Zebrafish" was published in 2010. Journal: PLoS One.

### Transmission electron microscopy (TEM)

Embryos injected with MOs were dechorionated at 8 hpf, fixed with 2% fresh paraformaldehyde and 2.5% glutaraldehyde in 0.1 M cacodylate buffer (pH = 7.4) at 8.5 hpf for 2 h at room temperature, washed by the same buffer, and then post-fixed with 1% OsO_4_ in the same buffer for 2 h on ice. They were then rinsed with distilled water, stained with 0.5% aqueous uranyl acetate overnight at room temperature, dehydrated with ethanol series then 100% acetone, and embedded in Spurr's low-viscosity embedding mixture (Electron Microscopy Sciences). Ultrathin sections were cut with diamond knives, double-stained with uranyl acetate and lead citrate, and examined with a Hitachi H-7650 transmission electron microscope (Toronto, Ontario, Canada).

### Ventral leading edge observations

Embryos injected with designated MOs and membrane-bound GFP-GAP43 messenger RNA (mRNA) were dechorionated and mounted in 1% low-melting-point (LMP) agarose (AMRESCO, Solon, OH) at 6.5 hpf. Embryos then were monitored in regions of the ventral leading edges under confocal microscope (TCS SP5, Leica Microsystems). Time-lapse images of suitable embryos were taken at 10-s intervals for 10 min.

### Cell tracing assay

Embryos were injected with 1% (w/v) caged Q-rhodamine dextran (Invitrogen, Carlsbad, CA) and 7.5 ng *cfl1* tMO_1_ dissolved in injection buffer mixed with 1% Q-rhodamine were injected into embryos at one cell stage. The embryos were grown in dark until 50% epiboly and immobilized at an injection through on a 50 mm 1% agar plate. To uncage Q-rhodamine, a beam of ultraviolet light through a DAPI filter set under an automatic upright microscope system (DM5000B, Leica Microsystems, Wetzlar, Germany) with a 40X water objective, was directed for 1∼3 s at the lateral blastoderm margin [33]. Both dark and bright field images were taken using a CoolSNAP *fx* charge-coupled device (CCD) camera (Roper Scientific, Tucson, AZ). Images were collected and analyzed using Simple PCI Imagine System software (Compix, Sewickley, PA).

The article "Loss of Cofilin 1 Disturbs Actin Dynamics, Adhesion between Enveloping and Deep Cell Layers and Cell Movements during Gastrulation in Zebrafish" was published in 2010. Journal: PLoS One.

### Cell protrusion assay

Embryos injected with MOs were dechorionated and mounted in 0.8% LMP agarose at the sphere stage for lateral cell observations, or at the shield stage for prechordal plate cell observations. Differential interference contrast (DIC) optical time-lapse images were acquired and analyzed by the Simple PCI Imagine System software for 15 min at 15-s intervals under the DM5000B system with a 40X water immersion objective.

### Cell transplantation assay

Donor embryos were injected with dextran, tetramethylrhodamine (10,000 MW, anionic, fixable, Invitrogen) and designated MOs. After the 1k-cell stage, host embryos were dechorionated by 10 mg/mL protease (Sigma, St. Louis, MO) and mounted in 0.8% LMP agarose. Cells from donor embryos were then transplanted into host embryos at approximately the sphere stage using CellTram vario (Eppendorf, Hamburg, Germany). The single focal plane time-lapse recordings of transplanted cells were collected at 30-s intervals for 1 h during late gastrulation (at 7∼9 hpf) using the 40x water-immersion objective under the DM5000B system and analyzed by the SimplePCI Imagine System software. The transplanted cells were also observed under confocal microscopy (TCS SP5, Leica Microsystems) and 10-min movies were recorded at 15-s intervals.

## Supporting Information

Movie S1 **Time‐lapse confocal imaging of dorsolateral cell migration in StdMO‐injected embryo.** Embryos were also injected with membrane‐bound green fluorescent protein mRNA to reveal the membrane. Shown here is a 10‐min movie at 15‐s intervals time‐lapse confocal image sequence. The cells were migrating toward the vegetal pole.
(MOV)

Movie S2 **Time‐lapse confocal imaging of dorsolateral cell migration in *cfl1* tMO1‐injected embryo.** Embryos were also injected with membrane‐bound green fluorescent protein mRNA to reveal the membrane. Shown here is a 10‐min movie at 15‐s intervals time‐lapse confocal image sequence. The cells were migrating toward the vegetal pole.
(MOV)

Movie S3 **Time‐lapse imaging of pseudopod formation in involuting lateral cells of a wild type embryo injected with StdMO.** Shown here is a 15‐min DIC time‐lapse image sequence of a StdMO‐injected embryo. The lateral cells were migrating toward the animal pole on the top.
(MOV)

Movie S4 **Time‐lapse imaging of pseudopod formation in involuting lateral cells of a wild type embryo injected with *cfl1* tMO1.** Shown here is a 15‐min DIC time‐lapse image sequence of a *cfl1* tMO_1_‐injected embryo. The lateral cells were migrating toward the animal pole on the top.
(MOV)

Movie S5 **Time‐lapse imaging of pseudopod formation in involuting prechordal plate cells of a wild type embryo injected with StdMO.** Shown here is a 15‐min movie at 15‐s intervals DIC time‐lapse image sequence of a StdMO‐injected embryo. The prechordal plate cells were migrating anteriorly to the left.
(MOV)

Movie S6 **Time‐lapse imaging of pseudopod formation in involuting prechordal plate cells of a wild type embryo injected with *cfl1* tMO1.** Shown here is a 15‐min movie at 15‐s intervals DIC time‐lapse image sequence of a *cfl1* tMO_1_‐injected embryo. The prechordal plate cells were migrating anteriorly to the left top corner.
(MOV)

Movie S7 **Time‐lapse confocal imaging of Std‐MO‐treated cells transplanted into an untreated wild type embryo.** Shown here is a 10‐min movie at 15‐s intervals time‐lapse confocal image sequence. The transplanted cells were migrating toward the vegetal pole.
(MOV)

Movie S8 **Time‐lapse confocal imaging of *cfl1* tMO1‐treated cells transplanted into an untreated wild type embryo.** Shown here is a 10‐min movie at 15‐s intervals time‐lapse confocal image sequence. The transplanted cells were migrating toward the vegetal pole.
(MOV)

Movie S9 **Time‐lapse confocal imaging of Std‐MO‐treated cells transplanted into a *cfl1* tMO1‐injected embryo.** Shown here is a 10‐min movie at 15‐s intervals time‐lapse confocal image sequence. The transplanted cells were migrating toward the vegetal pole.
(MOV)

Movie S10 **Time‐lapse confocal imaging of *cfl1* tMO1‐treated cells transplanted into a *cfl1* tMO1‐injected embryo.** Shown here is a 10‐min movie at 15‐s intervals time‐lapse confocal image sequence. The transplanted cells were migrating toward the vegetal pole.
(MOV)
